The article "The Application of Artificial Intelligence in Football Risk Prediction" was retracted in 2023. Reasons: unreliable results or conclusions; concerns about the data; concerns about the peer review; concerns about the citations.

# The Application of Artificial Intelligence in Football Risk Prediction

**DOI:** 10.1155/2022/6996134

**Published:** 2022-06-13

**Authors:** Jinyu Qiao

**Affiliations:** Sports Department, Puyang Vocational & Technical College, Puyang 457000, Henan, China

## Abstract

Football is the most popular sports in the World, with an estimated global following of 4.0 billion fans worldwide. Football draws attention from people of various age groups. The result of the game only decides the performance of the team and individual players. The player has to train smarter to avoid a career-ending injury. Sports have also entered into the new era of artificial intelligence as any industry. Artificial intelligence (AI) in football acts like a teammate to the players and also plays the role of an assistant coach. The coach uses artificial intelligence and incorporates it into the traditional way of training. The Football Associations have already implemented sensors to collect data in the form of technologies such as Video Assistant Referee and Goal Line Technology. Additionally, the quality of the players and the coaches is improved with smart technological implementation. This technology itself incorporates the utilization of smart technologies for data acquisition using sensor networks and an intelligent data analysis. The proposed algorithm is compared with the fuzzy logic model (FLM) and found that it is 7.2% of higher risk predication by the proposed model than the existing.

## 1. Introduction

Due to the enormous abundance of data and the approaching need to turn this data into valuable information and practical solutions, artificial intelligence (AI) has been a hot issue among researchers and practitioners for many years. However, the use of data is still in its infancy in several areas, such as sports [1]. In sports, as in many other sectors, automated data analysis is becoming increasingly important and rapidly developing. As a result of comprehensive data analysis, sport science practitioners and researchers can make better training and competition decisions [2]. Modern data-driven statistical methods have become a hot topic in sports science because they fill in the gaps left by more traditional statistical methods. Expertise in integrating statistical and computational tools into bigger frameworks and solving specific problems is necessary in data science [3]. Analyzing and interpreting data requires an understanding of its context, an appreciation of the responsibility that comes with accessing private and public data, as well as an ability to effectively communicate the findings of a dataset [4]. Algorithms can be improved and tinkered with the help of learning models in order to help athletes and sports professionals make better judgments and get useful advice. Both supervised and unsupervised learning may be achieved using these techniques (e.g., clustering) [5]. For example, one type of supervised learning requires both input and output data, while the other does not. Data science is being used in a wide range of industries, including social networking and streaming services, healthcare, manufacture, educational programmes, financial modelling, policing, and marketing are all included in this category [6]. It has also been suggested that the use of science and technology to improve sports performance has a bright future in our field. The R&D departments of the world's largest technological firms could generate sports innovation, introduction, and enhancement. Sport professionals employ data (physical, technical, and tactical) and their expert judgment while making decisions concerning athletes in a fast-paced context [7].

The article "The Application of Artificial Intelligence in Football Risk Prediction" was retracted in 2023. Reasons: unreliable results or conclusions; concerns about the data; concerns about the peer review; concerns about the citations.

Nevertheless, for those in the sports medicine and science professions, success in team sports requires making decisions based on evidence in order to minimize injury risk and maximize the performance of athletes. Players, coaches/managers, and other members of the sports community can benefit greatly from research and innovation [8]. Because of this, we must provide solutions that have a direct influence on their daily life. A major issue in sports medicine is the need to be able to accurately forecast both injury risk and performance. They may prescribe training that will generate the best results with the least chance of injury because they have had years of experience with the sport they are coaching [9]. When it comes to developing training programmes using scientific methods, however, modern approaches are warranted. Using new statistical methods from artificial intelligence could help prevent injuries and enhance automobile models (AI). While some consider it the “world's first sport,” many others consider football to be an all-encompassing and universally loved hobby. Since the sport is so popular and competitive, participants are more prone to suffer from a variety of ailments and strains as a result [10]. The phrase “sports injury” encompasses a wide range of injuries that are associated to sports. Athletes' sports training methods, sports strategy, and athletes' sports environments all have a role in the likelihood of sports-related injuries. There is harm to both the human body's motor system and the blood vessels and neurological system [11]. Players in football face a high risk of injury because of the frequency and severity of their injuries. It has been shown that football players' knee injuries are the most common in the sport and have an enormous effect on their physiological makeup. The most common sports injuries in football are to the knees, including athlete's tibia joint soreness, tendonitis, sacral syndrome, quadriceps tendinitis, and athlete's knee surrounding bursitis [12]. It is referred to as the “cognitive risk” of knee damage because of the discrepancy between trainers' subjective and objective assessments of the risk. Based on a player's performance and the severity of their consequences, it is possible to predict whether or not they may suffer knee ligament damage while playing [13]. Football players' ability to compete is significantly impacted by sports injuries. There are a lot of athletes that suffer from knee problems, which are both common and serious. During training and competition, football players are hindered by knee injuries. In football, consistent practise and competition were ineffective in enhancing a player's competitiveness. Because of knee injuries that are too frequent, they may also end a player's athletic career [14]. To avoid training-related knee injuries, it is necessary to model the knee joint. As a result of this problem, a number of effective forecasting algorithms have been developed. The researcher proposes a healthcare data-based knee injury prediction algorithm for football players [15]. During a football game, researchers surveyed more than 800 participants with questionnaires. The causes of the players' knee injuries during this football game are then determined. Analytical results are used to forecast knee joint injuries. Researchers have found that knee joint problems in football are largely due to their particular shape [16]. The athlete's technical ability, awareness of personal safety, and level of activity are all influenced by external influences during practice. During this time, the athlete is also receiving medical attention [17]. As a result of poor warm-up preparation, poor technique, and lack of awareness, football players are more likely to suffer knee injuries than other athletes, according to an analysis of healthcare data. This data analysis may put the knee joints of players at risk, according to research studies. This method can be used to some extent to forecast the likelihood of knee damage in football players [18]. It is difficult to know for sure how to avoid or treat future knee problems because there are still a lot of unknowns.

The article "The Application of Artificial Intelligence in Football Risk Prediction" was retracted in 2023. Reasons: unreliable results or conclusions; concerns about the data; concerns about the peer review; concerns about the citations.

In the literature, an algorithm has been developed for predicting the likelihood of knee joint damage in football players [19]. A stratified cluster sample method was used to gather information on the injuries suffered by 5,000 spectators at a national football match. Athletes' gender, injury time, injury site, injury kind, and cause are all recorded in a survey [20]. According to a study, 53.9 percent of football players had been injured. In athletics, the knee is the most frequently injured joint. The most common knee injuries are abrasions, sprains, contusions, and strains. 27.3 percent of these injuries are attributed to male football players, while 26.7 percent are attributed to female athletes [21]. There are 57.5 percent of all knee problems that can be traced back to a faulty warm-up regimen. 40 percent of the time athletes commit technical errors, and 43 percent of the time athletes are motivated by their own personal physique. The findings of a stratified cluster sample study suggest that the knee joints of football players could be injured. Predictions made by the algorithm are not always accurate [22].

When it comes to predicting knee injuries, a longitudinal monitoring study of 200 Shandong Province football players was conducted to document all knee injuries as well as the conditions that affect athlete training [23]. It is only orthopaedic surgeons that can accurately diagnose a knee injury in an athlete. Among athletes in different grades and years, this study compares the hazard ratio of knee joint injury [24]. A total of 100 athletes were injured throughout the game, with 27 cases of acute knee trauma, 19 cases of preexisting knee ailments, and 11 cases of knee strains. Recent years have seen significant advancements in swarm intelligence, machine learning predictions, and evolutionary methods. The Knapsack problem, the scheduling of ‘m' jobs on ‘n' resources, the travelling salesmen problem, the subset sum problem, and stopping problems are other examples [25]. Real-world prediction and classification problems can be solved using deep and machine learning. As time goes on, the algorithms are improving in performance. To overcome the shortcomings of existing knee injury prediction algorithms, an intelligent knee injury prediction method is given. Experiments have shown that this technique can increase both the accuracy of knee injury prediction and its precondition in football players [26]. This study focused on evaluating the risk prediction in football using artificial intelligence technique.

## 2. Proposed Method

In the traditional coaching style, with the help of the knowledge shared by the coach and the frequent self-check of one's own body during training and game, the players had to predict whether they might receive an injury shortly. Nowadays, in top-level teams, the players are monitored with the help of tight tops worn under the jersey, which contains GPS, an accelerometer, gyroscope, and related sensors. These sensors track the player's speed, distance covered, and heart rate during the training session and matches. This process is repeated indefinitely, and these data are fed into machine learning to detect a player's current status and play pattern. AI predicts that a player may get injured in a few days from this data. Injuries are caused due to too much pressure put on the body, frequency of training, and intensity of exercise. Coaches will monitor the condition of players when scheduling training sessions. Coaches can now calculate more precisely the probability that a player will get injured during the next match or somewhere near in the coming days.

The article "The Application of Artificial Intelligence in Football Risk Prediction" was retracted in 2023. Reasons: unreliable results or conclusions; concerns about the data; concerns about the peer review; concerns about the citations.

The football stadium is built in a smart city concept with the usage of WSN. Injuries during training and match are more common in football matches. These injuries are due to the high-speed action combined with running. The most common injuries are traumatic injuries, overuse injuries, heat injuries, and concussions. In worst cases, players are prone to end their careers due to injury. The processes involved in football risk prediction are as follows:

1. Players with AI-assisted wearables: players wear tight tops with sensors, accelerometers, gyroscopes, GPS, etc., to monitor the heart rate, speed, and distance covered. The team and coach will monitor these data in every training and game session. Research is introducing AI-assisted helmets to avoid head injuries and collect data.
2. Monitoring players' movements and record: the player's speed and the distance he covers in the game session are monitored. The dynamics of the player, i.e., fast and hard accelerations are recorded as well. The shot speeds, ball handling, and pass possession completion rates are essential in the data set.
3. AI predicted upcoming injury: the collected dataset predicts that a player may get injured in a few days. Injuries are caused by too much pressure put on the body, frequency of training, and intensity of exercise. The prediction will be very much valuable for the team. When a key player gets injured, the whole team will suffer. It may also need to lose the match.
4. Rest given to player: proper rest is given to the player after the identification process by the AI. The player will recover and heal fully in a medically instructed period. This considerably reduces the players getting injured, which has two disadvantages. The injured player may lose the chance to play the series or, in worst cases, ends up the career due to injury and affects the game if he is the leading player.
5. Resume to training and match: the player will resume training and game after the medically instructed recovery time. This time the training will be nominal and moderate to avoid risks. Again the data will be taken and checked. This checking ensures the safety of the players.

The article "The Application of Artificial Intelligence in Football Risk Prediction" was retracted in 2023. Reasons: unreliable results or conclusions; concerns about the data; concerns about the peer review; concerns about the citations.

Besides these, life-saving IoT is also implemented for avoiding the major risk. It is highly recommended to carry sensor devices for predicting risk.

Thus, AI plays the role of a teammate and is more like an assistant to the coach, aids in avoiding injuries; it is also life-saving. Adapting to the new AI technology in a football game will also become a safe sport. The process of football risk identification and management is depicted in Figure 1. The data are collected with the aid of smart sensors attached to the training location that functions using intelligent wireless networking.

### 2.1. Proposed Work

The study assesses the use of machine learning in critical analysis of football risk prediction sports statistics using research methodology including scientific reports, audio/video analysis, research methods, and mathematical statistics. The suggested football risk prediction position here on issue action recognition as well as analysis system is divided into two parts that are interconnected. The underside position estimate analysis is used to identify the find a good in the first segment, which is used to extract the user's body position procedure from video. The analysis of the ANN machine algorithms here on space-time diagram seems to be the second component. Football risk prediction activity in the predefined classification is identified and extracted from fragmentation and performed in a viewpoint sequence. In comparison to traditional training, the other method seems to be a supplementary method to increase accuracy while correcting playmaker errors in a timely manner. The technique helps players' accurate technical errors, building muscle memory, and improve their skills. As AI techniques and implementations reach a wider audience, higher education confronts both an incredible opportunity. As WSN with AI techniques applied becomes more popular, higher education needs to face both a challenges and opportunities. While attempting to integrate many of the positive aspects of WSN with AI, education faces a number of challenges, including the development of standards and the provision of adequate guidance and support. It is proposed that viewer and shared recognition systems are two possible approaches to bridging the gap between these two civilizations while also mentioning instructional fears. The simplified workflow of the proposed system is shown in Figure 2.

Within the first process, users have used the variation among the statistical features over all frames around that one, *K*_*n*_, as the characteristic, that is also described as

(1) $$\begin{array}{c} \sum_{i=1}^{m}\Delta i,m_{i}\in m,m_{i}\neq u_{i}^{*}:d_{i}\left(m_{i}^{*},m_{-i}^{*}\right)>\sum_{i=1}^{m}d_{i}\left(m_{i},m_{-i}^{*}\right). \end{array}$$

Also, every player *i* can acquire about their utility for various modes *d*_*i*_(*n*_1_, *n*_2_,…, *n*_*m*_) of strategic approach. A Nash equilibrium point is a profile of {*m*_1_^*∗*^, *m*_2_^*∗*^,…, *m*_*m*_^*∗*^} ∈ *mm* strategy if no change in strategy by a player leads to high, low, etc. Various other players are represented by *Q* = (*Q*_1_, *Q*_2_,…, *Q*_*n*_). Based on time steps, the equation *P*_*ij* _ shows the prediction of every task across each resource. Make the assumption *D*_*n*_ which is the total amount of task bidding wars for the resource as that of the price with one resource at that time, and equation (2) is obtained:

(2) $$\begin{array}{c} Q_{h}=\frac{\sum_{i=0}^{P}\left|D_{n}\left(i\right)-D_{n-1}\left(i\right)\right|}{\text{Width}\cdot \text{Height}}>W_{y}, \end{array}$$

where *P* denotes its quantity of colour histogram, *Q*_*n*_ and *Q*_*n*−1_ represent the colour histograms of clips *n* with *n* − 1, respectively, equation (3), Width. Height represents the number of pixels in each frame, and *W*_*y*_ represents the thresholds for identifying a single maximum activity in a series of *K*_*h*_ deformation values.

(3) $$\begin{array}{c} A_{n}=\sum_{i=1}^{n-1}\frac{CQ_{n-1}}{Ci_{n-1}}\;\text{for }I-\text{frame}, \end{array}$$

where CQ, Ck, Ci, but Ci are the CBs not only for intracoded, forward predicted, and head back predicted frames but also for bidirectionally predicted frames, but rather *n* is the structure size:

(4) $$\begin{array}{c} A_{n}=\sum_{n=1}\frac{IP_{n}}{CN_{n}}\;\text{for }b\text{ frame}\text{.} \end{array}$$

Humans altered A by putting up a b-frame. A conceptualization to have more precise results equation (4) when the boundary takes place at I-frames:

(5) $$\begin{array}{c} A_{n}=\sum_{n=1}^{i}\frac{\left|CQ_{n}-Ck_{n}\right|}{Ci_{n}}\;\text{for }H\text{ frame}. \end{array}$$

In equation (5), involved thresholds to modifying the H-frame RFD appearance to decrease false alarms if *Ck*_*n*_ and *CQ*_*n*_ are both considerably greater than Bin. Examination of the frame developments are shown in the equations from (6)–(9):

(6) $$\begin{array}{c} Q_{n}\left(0\right)=\sum_{n-1}^{n}\text{if }\left(Ck_{n-1}-CN_{n-1}\right)>0, \end{array}$$

(7) $$\begin{array}{c} Q_{n}\left(1\right)=\sum_{n=1}^{n}\text{if }\left(Ck_{n}-CN_{n}\right)\times \sum_{n=1}^{n}\left(Ck_{n-1}-CN_{n-1}\right)\leq 0\;\text{for }H\text{ frame,} \end{array}$$

(8) $$\begin{array}{c} Q_{n}\left(0\right)=\;\sum_{n-1}^{n}\text{if }\left(Ck_{n}-CN_{n}\right)\;\times \sum_{n=1}\left(Ck_{n-1}-CN_{n-1}\right)>0\;\text{for }H\text{ frame,} \end{array}$$

(9) $$\begin{array}{c} m_{i}=\sum_{i=1}^{b}b_{1}m_{i}+b_{2}y_{i}+b_{3}. \end{array}$$

In equation (10), *Qs*_*i* _ and *Qy*_*i*_ are also the resampling constituents for a specific structuring element is represented:

(10) $$\begin{array}{c} Qy_{i}=\sum_{i=1}^{b}b_{4}m_{i}+b_{5}y_{i}+b_{6,}. \end{array}$$

The *b*_*i*_′*s* linear parameters we call interpolation linear parameters are denoted by *m*_*i*_ and *y*_*i*_ and seem to be the spots risk prediction of the CB's centroid. The row vector *h*_*i*_=(*m*_*i*_, *y*_*i*_, 1) is described. The coordinate matrix C is then generated for all blocks that are not marked as outliers by vertically concatenating the row vectors *h*_*i*_. W is a *Q* × 3 matrix because *M* is the number of macro blocks that are not marked as outliers. The vectors *d*_*m*_ and *d*_*y*_ are created by adding all of *m*_*i*_ with *y*_*i*_ for the HBs that are not identified as outliers. Finally, the linear interpolation parameters *P*_*m*_=(*P*_1_, *P*_2_, *P*_3_)^*T*^ with *P*_*y*_=(*P*_4_, *P*_5_, *P*_6_)^*T*^ are combined. Based on these equations, we can write *D*_*s*_=*WP*_*s*_ and *D*_*y*_=*WP*_*y*_, which are then computed for *P*_*x*_ and *P*_*y*_ using R's formation matrix. Following equations (11) and (12),

(11) $$\begin{array}{c} P_{m}=\sum_{m=1}^{T}{\left(W^{T}W\right)}^{-1}W^{T}D_{m}, \end{array}$$

(12) $$\begin{array}{c} P_{y}=\sum_{m=1}^{y}{\left(W^{T}W\right)}^{-1}W^{T}D_{y}. \end{array}$$

Camera's horizontal movement (CHM) is represented as

(13) $$\begin{array}{c} \text{CHM}=\frac{\sum_{i=0}^{m}P_{3i}}{W}+\int {\left(W^{T}W\right)}^{-1}W^{T}D_{y}. \end{array}$$

Camera's vertical movement (CVM) is specified as

(14) $$\begin{array}{c} \text{CVM}=\frac{\sum_{i=0}^{m}P_{6i}}{W}-\int {\left(W^{T}W\right)}^{-1}W^{T}D_{y}. \end{array}$$

Camera's Zoom (CZD): the above features are defined as

(15) $$\begin{array}{c} \text{CZD}=\sum_{i=0}^{m}\frac{P_{1i}+P_{5i}}{2}+\int {\left(W^{T}W\right)}^{-1}W^{T}D_{y}. \end{array}$$

In equation (16), (*f*) represents the total number of images to obtain in the image-influenced outcome:

(16) $$\begin{array}{c} \text{Frequency }\left(f\right)=\sum 6495\times {\text{log}}_{10}\left(1+\frac{f}{900}\right). \end{array}$$

Frequency (*f*) is the sports risk prediction measurement unit of the normal frequency scale. The highest prevalence has a frequency spectrum of 0–30130 Hz and fixed frequency spacing for risk prediction is represented in the following equation:

(17) $$\begin{array}{c} m_{n}=\sqrt{\frac{2}{k}}\sum_{k=1}^{k}\left(\text{log}m_{k}\right)\sum_{n=1}^{n}\text{sin}\left[n\left(k-0.6\right)\frac{\pi }{k}\right],\;n=1,2,\ldots ,m. \end{array}$$

The energy measures the changes in the speech signals. With audio recordings *m*_*n*_, where *n*=1,2,…, *m*, 0.6 is specified for the energy and is calculated as the log of the frequency components and using

(18) $$\begin{array}{c} d=\text{log}\sum_{k=1}^{k}m_{n}^{2}+\sum_{n=1}^{n}\text{sin}\left[n\left(k-0.6\right)\right]. \end{array}$$

The article "The Application of Artificial Intelligence in Football Risk Prediction" was retracted in 2023. Reasons: unreliable results or conclusions; concerns about the data; concerns about the peer review; concerns about the citations.

## 3. Results and Discussion

Figure 3 depicts how the ANN technique needs to perform data-level classification of different data types, filters those, as well as eliminates errors combined with the decision-making processes inside this procedure; second, it incorporates the characteristics of various types of athletes in risk prediction. Arrays of varying sorts are depicted, and their data are further distinguished. Furthermore, the quantity of the machine learning method used during the analysis of various football risk prediction training arrays varies, and it varies by type.

The continued rise of Internet offerings that can be classified as Wireless Sensor Network (WSN) with AI has triggered a huge interest in education. The numerical representation of the figure is represented in Table 1. From this table, it can be seen that the players are divided into two teams as Team A and Team B. Certain prediction categories such as risk prediction playing surface view, flight view, fast playing surface view, slow playing surface view, more than four fouls (penalty), in fast playing medium surface view, out-of-playing or close-up surface view, and others are considered. From the frequency analysis, it can be observed that, at certain categories, Team A outperforms Team B and vice versa.

In WSN with AI predicting football risk, there seem to be significant differences between higher education values and those found in the WSN with AI collective in terms of classification frequency for level 1 and level 2 categories. WSN and AI methods have several key characteristics in common. The first is democracy; the second is that it is based on an undersurface approach; also, the third, in terms of education, is that they will be engaging.

Figure 4 depicts the variables that not only have a greater impact on the sports training procedure besides integrating several neural network (WSN with AI) analysis methodologies but also selected high-resolution elements to create a good connection between detection and risk prediction tracking and different dynamic performances. It has been discovered that sports have a low resolution difficulties during training and testing. They carried out a series of control trials to finalize not only the multifunctional implementation of various knowledge but also statistics.  Table 2 provides the numerical analytic report of the previous figure. From the table, it can be seen that analysis is performed on four major categories such as risk prediction training statistics, risk prediction testing statistics, football risk predication learning, and football risk prediction testing. The analysis is performed with the implementation of ANN algorithm and the metrics utilized are count, mean, standard deviation, and minimum and maximum values.

The article "The Application of Artificial Intelligence in Football Risk Prediction" was retracted in 2023. Reasons: unreliable results or conclusions; concerns about the data; concerns about the peer review; concerns about the citations.

In Figure 5, the implementation of ANN algorithms in sports matches was discovered, but it was discovered that qualitative difference conceptual methodology is presented solely on the machine learning method and was used for information processing within having trained data analysis correlation of football risk prediction sports, but it was discovered that this method has seemed to have more benefits. WSN with AI adds to this procedure the removal of a clarifier significant role played by financial intermediary that was previously a necessary part of the original design.

Table 3 represents the performance result analysis for monitoring the football risk prediction using intelligent wireless networking. The metrics utilized for analysis is count, mean, standard deviation, minimum, and maximum, by taking the analysis parameter as vertical (max), vertical (max reach), and vertical (no step).

In Figure 6, the technique of football risk prediction players willingness to acknowledge different styles of trainings was attempted to introduce, as well as the particle swarm technique for optimization evaluation and an ANN algorithm based solely on random sampling matrix. The results from Table 4 show that the algorithm can help with the possible solution of sports players' gait recognition while moving fluidly, though at the expense of selective recognition accuracy. The proposed model assumes that the gap between different seemingly disparate worlds might be bridged after considering the various learning education and WSN with AI, as well as some of the potential conflicts. This research focuses on the potential role of training and physical exercises which has to be given to the players who may need to change, with other bridging techniques, such as the development of appropriate technologies, which will undoubtedly be required.

The results in Figure 7 show that its algorithm could well solve the problem of sports football risk prediction pedestrian detection through fluid movement, albeit at the expense of insufficient recognition accuracy. The authors proposed a modified method for deflection gait region detection on ant colony as well as ANN algorithms to improve recognition accuracy. It is of high quality and can recognize a football risk prediction and take a step while training. This can be used to calculate the rotational movement of the heel joint and the training effect.

The article "The Application of Artificial Intelligence in Football Risk Prediction" was retracted in 2023. Reasons: unreliable results or conclusions; concerns about the data; concerns about the peer review; concerns about the citations.

Almost all of the discussion among trainers about WSN with AI revolves around quality and the metrics to be considered for reduced risk in the football training and during game event. A set that allows the players and the coaches to share learning algorithms could aid in resolving this issue by providing an educational structure based on resources that can then be altered. Football risk prediction may be able to close some of the contextual gaps that exist between WSN and AI, as well as higher education. From Table 5, it can be seen that the proposed ANN algorithm is compared with the existing fuzzy logic to predict the risk of the players during training and also at the time of an event. The performance analysis is performed on the basis of ground truth, recall, and precision. In all these analyses, it is observed that the ANN has received a precision of 99.6%; it means that exact classification is higher. The football risk prediction is 7.2% higher in comparison to the existing algorithm.

## 4. Conclusions

Using scientific reports, audio/video analysis, research methods, and mathematical statistics, the study examines the use of machine learning in critical analysis of football risk prediction. The study used ANN algorithm with WSN technologies for evaluating the risk of the players during training and time of an event. The study results revealed that the ANN model works well than existing algorithms. In addition to this, the algorithm has high precision of 99.6%. This research is carried out only on the basis of technological involvement and has not collected data about the experiences by the coaches or players. Besides the technology utilization, the player should obtain detailed information from the earlier players and the corresponding scenarios. In this context, the data can be collected and incorporated in the training process of the player to get wider knowledge about the safer mode to play games, maintain health conditions, and so on, as future enhancement. Additionally, evaluation in the prediction of risk injury at joints can also be focused.

## Figures and Tables

**Figure 1:** Architecture of AI in football risk prediction.

**Figure 2:** Overall workflow of the proposed system.

**Figure 3:** Football risk prediction using WSN and AI Classification frequencies for levels 1 and level 2.

**Figure 4:** Performance analysis for football risk prediction using machine learning WSN with AI techniques.

The article "The Application of Artificial Intelligence in Football Risk Prediction" was retracted in 2023. Reasons: unreliable results or conclusions; concerns about the data; concerns about the peer review; concerns about the citations.

**Figure 5:** ANN algorithm with performance analysis for vertical risk prediction in football using AI with the machine learning method.

**Figure 6:** In the machine learning method, ANN algorithm uses performance analysis for leg (Width) and agility then sprint of football risk prediction.

**Figure 7:** In the machine learning method, the ANN algorithm is used to predict football risk using overall performance analysis.

**Table 1:** WSN with AI for football risk prediction frequencies of categorization for level 1 and level 2 classifications' result.

Football risk prediction categories	Frequencies of analysis (%)	
	Team A	Team B
Risk prediction playing surface view	94.7	96.45
Flight view	98.6	95.34
Fast playing surface view	91.1	93.56
Slow playing surface view	86.5	88.43
More than four Fouls(Penalty)	96.4	85.34
In fast playing medium surface view	88.9	91.35
Out-of-playing (or) close-up surface view	85.8	79.4
Others	97.4	89.34

**Table 2:** Using AI with machine learning, perform a performance analysis to predict the height of a football player's risk.

	Risk prediction training statistics	Risk prediction testing statistics	Football risk prediction learning	Football risk prediction teaching
Count	64.05	64.03	64.03	64.07
Mean	68.83	76.16	86.85	98.45
Std	3.47	3.43	4.66	3.48
Min	69.23	76.57	63.07	86.53
Max	91.25	93.24	96.72	124.58

**Table 3:** ANN algorithm with performance result analysis monitoring for football risk prediction using AI.

	Vertical (max)	Vertical (max reach)	Vertical (no step)
Count	44.01	46.01	46.03
Mean	38.72	124.06	36.36
Std	3.74	4.9	4.56
Min	39.01	146.51	35.53
Max	48.03	157.04	37.55

**Table 4:** ANN algorithm with performance analysis for ground truth and recall, followed by precision of football risk prediction using machine learning technique result.

	Ground truth	Recall (%)	Precision (%)
Count	66.03	47.03	53.04
Mean	9.06	19.28	5.37
Std	4.44	2.51	3.12
Min	2.08	25.28	6.18

**Table 5:** Comparison result evaluation of football risk prediction in machine learning method result.

Performance	Ground truth	Recall (%)	Precision (%)
Risk prediction with ANN	31	93.5	99.6
Risk predication using fuzzy logic	52	95.7	92.4

## Data Availability

The data used to support the findings of the study can be obtained from the corresponding author upon request.
